The article "Upper-Limb Muscle Synergy Features in Human-Robot Interaction with Circle-Drawing Movements" was published in 2021. Journal: Appl Bionics Biomech.

# Upper-Limb Muscle Synergy Features in Human-Robot Interaction with Circle-Drawing Movements

**DOI:** 10.1155/2021/8850785

**Published:** 2021-09-14

**Authors:** Cheng Wang, Shutao Zhang, Jingyan Hu, Zhejing Huang, Changcheng Shi

**Affiliations:** ^1^Emergency Trauma Surgical Department, Ningbo First Hospital, Ningbo, Zhejiang 315010, China; ^2^Cixi Institute of Biomedical Engineering, Ningbo Institute of Materials Technology and Engineering, Chinese Academy of Sciences, Ningbo, Zhejiang 315300, China; ^3^Rehabilitation Department, Ningbo Yinzhou No. 2 Hospital, Ningbo, Zhejiang 315192, China

## Abstract

The upper-limb rehabilitation robots can be developed as an efficient tool for motor function assessments. Circle-drawing has been used as a specific task for robot-based motor function measurement. The upper-limb movement-related kinematic and kinetic parameters measured by motion and force sensors embedded in the rehabilitation robots have been widely studied. However, the muscle synergies characterized by multiple surface electromyographic (sEMG) signals in upper limbs during human-robot interaction (HRI) with circle-drawing movements are rarely investigated. In this research, the robot-assisted and constrained circle-drawing movements for upper limb were used to increase the consistency of muscle synergy features. Both clockwise and counterclockwise circle-drawing tasks were implemented by all healthy subjects using right hands. The sEMG signals were recorded from six muscles in upper limb, and nonnegative matrix factorization (NMF) analysis was utilized to obtain muscle synergy information. Both synergy pattern and activation coefficient were calculated to represent the spatial and temporal features of muscle synergies, respectively. The results obtained from the experimental study confirmed that high structural similarity of muscle synergies was found among the subjects during HRI with circle-drawing movement by healthy subjects, which indicates healthy people may share a common underlying muscle control mechanism during constrained upper-limb circle-drawing movement. This study indicates the muscle synergy analysis during the HRI with constrained circle-drawing movement could be considered as a task for upper-limb motor function assessment.

## 1. Introduction

The upper-limb rehabilitation robots can provide continuously haptic assistance or resistance to stroke patients with motor impairments in order to help them restore the motor function of upper limbs [1]. Since it was early developed in the 1990s [2], the upper-limb rehabilitation robot has been gradually recognized as an effective medical device which could assist some stroke patients to restore or improve their motor functions of upper limbs [3]. Besides training, rehabilitation robots have a potential to be considered as an objective rehabilitation assessment tool due to a plenty of sensors could be integrated into robotic systems and motor functions (i.e., range of motion, force, velocity, and muscle tone and strength) of upper limbs could be quantitatively detected and analyzed [4, 5]. Those assessment results can be obtained after training and provided to physicians locally or remotely in order to optimize the rehabilitation therapy. Moreover, some assessment results are also analyzed during the training process and provided to patients in order to visualize the rehabilitation progresses and enhance their training motivation.

Circle-drawing is one of typical human-robot interaction (HRI) tasks which are widely applied to quantitatively evaluate upper-limb motor function by using rehabilitation robots [5]. The ability to accurately implement this movement task is related to coordination of both elbow and shoulder joints. Therefore, circle-drawing-related kinematic (i.e., roundness, area, averaged speed, and jerk) and kinetic (HRI force) parameters measured by motion and force sensors embedded in the rehabilitation robots have been widely studied as the potential assessment metrics for upper-limb motor functions [4, 6, 7]. However, the muscle synergies characterized by multiple surface electromyographic (sEMG) signals in upper limbs during HRI with circle-drawing movements are rarely investigated.

Tropea et al. compared the muscle synergies of upper limbs in stroke patients and healthy subjects and observed that the difference can reflect the functional deficit induced by the neural damages [8]. Scano et al. clustered the muscle synergies of stroke patients into five groups and found a deep characterization and relationship with clinical assessment methods [9]. The previous studies strongly suggested that muscle synergy analysis may be a potentially promising method for assessing motor function stroke patients. However, it remains unclear whether the consistency of normal or abnormal muscle synergy patterns in upper limbs for stroke patients is good enough for rehabilitation assessments. The main challenge is the multiple degree-of-freedom and redundancy for upper-limb movements, which may cause a large variation of muscular activation patterns.

Hence, in this study, the end-effector upper-limb rehabilitation robot (EULRR) which was developed in the lab was used as a tool to assist and confine the circle-drawing movements and measure the outcome of HRI tasks. The robot-assisted and constrained circle-drawing tasks for upper-limbs movement were used to increase the consistency of muscle synergy features. Both clockwise and counterclockwise circle-drawing tasks were implemented by all healthy subjects using right hands. The sEMG signals were recorded from six muscles in upper limb, and nonnegative matrix factorization (NMF) analysis was utilized to obtain muscle synergy information. Both synergy pattern and activation coefficient were calculated to represent the spatial and temporal features of muscle synergies, respectively. Reconstructed sEMG data were compared with the raw data in order to verify the effectiveness of NMF algorithm. The muscle synergy features of upper limb in HRI with two directions of circle-drawing movements were analyzed, and the consistency of muscular activation patterns was discussed.

## 2. Methods

### 2.1. Participants

Twelve healthy adults (10 males and 2 females and with average ages of 25 ± 1 years old) and two stroke patients (2 females, 67 and 39 years old, Brunnstrom stages III and IV) were involved in this study, who are all right-hand dominant, with no known neurological diseases, no muscular or skeletal impairments history of the upper limbs and the trunks, and no functional abnormalities. Before starting the experimentations, all the subjects signed an informed consent. The study was approved by the Ningbo Institute of Materials Technology & Engineering, Chinese Academy of Sciences. Informed consent was acquired from each subject.

### 2.2. EULRR System and sEMG Acquisition Device

The EULRR system mainly consists of motor, belt, reducer, frame, rocker, sensor, and a tray with a grip in space coordinates. The system has 5DOF in total: the rocker moves along the three axes; the rotation DOF of tray turns around *Z*-axis and *Y*-axis. The movement of *X*/*Y* direction is transmitted to the reducer by the *X*/*Y* shaft motor through the belt pulley and then transmitted to the frame by the reducer. The movement of *Z* direction is transmitted by the Z shaft motor through the pulley to the inside of the screw [10]. A 6-axis force/torque sensor is attached between the tray and the end of rocker to measure the force/torque exerted by the subjects. sEMG signal acquisition equipment uses TRIGNO wireless sEMG system (Delsys Inc., Massachusetts, USA) which has 16 4-channel sEMG and acceleration acquisition sensor, wireless transmission range is up to 20 m, sensor delay is less than 500 *μ*s (less than a sampling period), sEMG signal sampling rate is about 2000 Hz, baseline noise is less than 750 nV, it has 16-bit signal resolution, and sensor electrode is Ag-AgCl electrode with high conduction efficiency.

### 2.3. Upper-Limb Circle-Drawing Movement Tasks

After the sEMG electrode placement, the participants were asked to sit on the left side of the EULRR system and carried out all the tasks by using their right hands in the horizontal plane, as shown in Figure 1. In order to avoid unnecessary muscle compensation, they were informed to keep trunk steady and only use the upper limbs to complete the full circle-drawing movement by moving the joystick of EULRR, which constrained the circle radius of 10 cm. All subjects were instructed to carry out a series of trials (10 times per task). Subjects were asked to perform ten counterclockwise and clockwise circle-drawing movements from the start point arranged along the circular trajectory in a horizontal plane by holding a handle of joystick with a self-comfortable speed in different directions. Before starting the experiment, subjects performed a simple learning process under the guidance of instructors in order to complete the tasks smoothly.

### 2.4. sEMG Data Acquisition

During the circle-drawing tasks, the sEMG signals were recorded from six upper-limb muscles including anterior deltoid (AD), posterior deltoid (PD), biceps brachii (BB), triceps brachii (TB), flexor carpi radialis (FCR), and extensor carpi radialis (ECR). Electrodes were placed in accordance with the guidelines of sEMG for noninvasive assessment of muscles (SENIAM) [11]. Each recorded site was cleaned with alcohol and scrub cream before placing the electrodes. All the data were collected at the sampling rate of 2000 Hz.

### 2.5. Muscle Synergy Analysis

The collected sEMG signals were preprocessed according to the following steps before extracting muscle synergies: band-pass-filtering (20-400 Hz), subtracting signal mean values to remove direct current offsets, then rectified, and enveloped. Each row of the preprocessed sEMG matrix (*V*_*m*×*t*_, where *m* is the number of muscles and *t* is the recorded time) [12] was normalized with respect to its submaximal [13] and sampled into 1000 points. Because we rectified the EMG data, all components of the synergy are nonnegative is reasonable. NMF algorithm [12, 14] was chosen here to extract synergy pattern matrix *W*_*m*×*r*_ and activation coefficient matrix *H*_*r*×*n*_. So the synergy decomposition as the equation *V*_*m*×*n*_ = *W*_*m*×*r*_ × *H*_*r*×*n*_. A vector of *W*_*m*×*r*_ represents the relative weighting of muscles in each module, and the coefficient *H*_*r*×*n*_ represents the neural command that specifies how much each synergy will contribute to a total muscular activity pattern [15]. During the extraction, the number of synergy vector (*r*) was increased successively from one to six, and for each iteration of *r*, the NMF was repeated 20 times, and the repetition with the lowest residuals of reconstruction was selected.

Various methods have been used to determine the appropriate number of muscle synergies underlying a given dataset [16, 17]. The criterion of variance account for (VAF) [18–20] was adopted here in the following equation:

(1) $$\begin{array}{c} \text{VAF}=1-\frac{\sum_{i,j}{\left(V-V_{r}\right)}_{ij}^{2}}{\sum_{i,j}{V_{ij}}^{2}}, \end{array}$$

in which *V*_*r*_ is the reconstructed EMG matrix and the *V* is the initial EMG matrix. The number of synergy vectors (*N*) that sufficiently recaptured the original EMGs was then defined as the minimum number (*r*) when VAF exceeded 90% in more than half of the subjects in both groups. We checked the goodness of reconstruction of global and individual muscle's EMG at *N* synergy components, which is sensitive to both shape and amplitude of the signals [21].

In summary, the muscle synergy features were analyzed in different movement directions of circle-drawing during human-robot interaction in healthy and stroke subjects. This study mainly includes sEMG data collection during circle-drawing movement with the EULRR assisted, sEMG data preprocessing, and muscle synergy extraction and analysis. The first two parts can be used to obtain the processed sEMG signals. The muscle synergy features can be obtained by analyzing those processed sEMG data. The procedure of sEMG data preprocessing and muscle synergy analysis is shown in Figure 2.

## 3. Results

### 3.1. sEMG Results during Circle-Drawing Movement

The mean and normalized sEMG signal envelopes of 10 times of counterclockwise and circle-drawing movements are shown in Figure 3. The sEMG features in the process of HRI with circle-drawing movements were analyzed. The sEMG result for the counterclockwise circle-drawing movements is shown in Figure 3(a). Firstly, the BB and TB were activated in pairs and showed a negative correlation, which might indicate that TB contraction (relaxation) and BB relaxation (contraction) happened simultaneously and BB was activated slightly earlier at temporal domain. Secondly, the AD and PD were activated in pairs and showed a negative correlation. PD was activated slightly earlier at temporal domain. The sEMG result for the clockwise circle-drawing movements is shown in Figure 3(b). Firstly, the BB and TB were activated in pairs and showed a negative correlation. TB was activated slightly earlier at temporal domain. Secondly, the AD and PD were activated in pairs and showed a negative correlation. AD was activated slightly earlier at temporal domain.

### 3.2. The Results of Muscle Synergy Analysis

In the current study, we used VAF > 90% as the threshold to determine the number of muscle synergies. The mean VAF of all healthy subjects' 10 times circle-drawing movement demonstrated three muscle synergies can be appropriate for the sEMG data analysis. In Figure 4, the black solid curves represent the raw sEMG data, and the blue dotted line represents the reconstructed sEMG data. It can be seen that three types of muscle synergies were sufficient to reconstruct the original sEMG signal. According to the analysis on two stroke patients' data, two muscle synergies can be extracted from the raw sEMG data.

We used the model of time-invariant synergies to extract the muscle synergies [22]. A typical muscle synergy analysis result of counterclockwise circle-drawing movement tasks by healthy subjects is shown in Figure 5. The *W* represents synergy patterns, and *H* represents activation coefficients, and targeted muscle numbers 1-6 represent AD, PD, BB, TB, FCR, and ECR, respectively. The results demonstrated that the first synergy pattern mainly includes AD, and the corresponding activation coefficients were mainly activated at the ending of movements for all subjects. The second synergy pattern mainly includes BB, FCR, and ECR; meanwhile, the corresponding activation coefficients were mainly activated at the beginning of movements. The third synergy pattern mainly includes PD and TB; meanwhile, the corresponding activation coefficients were mainly activated at the middle process of movements.

Figure 6 shows a typical muscle synergy analysis result for clockwise circle-drawing movements conducted by the healthy subjects. The results indicated the first synergy pattern includes AD, and the corresponding activation coefficients were mainly activated at the ending of movements. The second synergy pattern mainly includes BB, FCR, and ECR; meanwhile, the corresponding activation coefficients were mainly activated at the middle process of movements. The third synergy pattern includes PD and TB; meanwhile, the activation coefficients were mainly activated at the beginning of movements.

Figure 7 shows a typical muscle synergy analysis result for counterclockwise circle-drawing movements implemented by stroke subjects. The first muscle synergy pattern includes AD, BB, and FCR which are all flexion muscles, and the corresponding activation coefficients were mainly activated at the ending of movements. The second muscle synergy pattern includes PD, TB, and ECR which are all extensor muscles, and the corresponding activation coefficients were activated from the beginning to the middle processes of movements. Compared to the results for the healthy subjects, the curve of activation coefficients for stroke patients has four peaks which might be induced by impaired muscular function of patients.

Figure 8 shows a typical muscle synergy analysis result for clockwise circle-drawing movements implemented by stroke subjects. The first muscle synergy pattern includes PD, TB, and ECR which are all extensor muscles, and the corresponding activation coefficients were mainly activated at the ending of movements. The second muscle synergy pattern includes BB, TB, FCR, and ECR; meanwhile, the corresponding activation coefficients were activated at the beginning of movements.

## 4. Discussion

Upper-limb rehabilitation robot could provide high-intensity, repetitive, task-specific, and interactive exercises for stroke patients. The robot could be effective to achieve the desired training functions, informing the subject to complete the task as well as enabling them to reduce unnecessary muscle activation [23]. Besides the training, the rehabilitation robot also can be developed as an efficient assessment tool for patients' upper-limb motor functions [24].

The structure of muscle synergy for a specific task may contain useful information on the residual ability of neuromuscular control in the poststroke patients. Stroke patients often have upper-limb problems due to abnormally high spasticity of muscles in the shoulder and elbow joints [25, 26]. Circle-drawing movement requires the coordination of both shoulder and elbow joints with multijoint movements. This task can be considered as a kind of task-specific, rhythmic, interactive training as well as an objective, reliable means of monitoring the change progress of patient's upper-limb motor function. Regarding the clinical practice, some kinematic indexes including circle area and roundness can give useful objective information regarding arm function of stroke survivors [6]. During robot-assisted rehabilitation process, it needs to promote the patients' muscle synergy to enhance the biomechanical functions of patients' upper limbs. Muscle synergy is helpful to increase understanding of the mechanisms involved in restoration of upper-limb function poststroke patients.

In this study, the constrained circle-drawing movements for upper limb were used as a task for motor function assessment. The results obtained from the experimental studies confirmed that high structural similarity of muscle synergies was found among the healthy subjects during HRI with circle-drawing movement, indicating that the healthy people may share a common underlying muscle control mechanism during constrained upper-limb circle-drawing movement. It was found that the muscle activation patterns regarding counterclockwise and clockwise circle-drawing movements demonstrated a complementary mode, which indicated that the activation coefficients of muscle synergies may be affected by the moving directions.

The results of muscle synergy analysis for stroke patients demonstrated the number of muscle synergy decreases when compared with the healthy subjects. The similar phenomenon was also found by Cheung et al., and this reduction of synergy number may be due to the neural function changes after patients' cortical damage [19]. The activation coefficients of muscle synergy for stroke patients were also found to be different when compared with the healthy subjects. There were more peaks in the activation coefficient curve, especially during the HRI with counterclockwise circle-drawing movements. This feature of activation coefficients might be related to the abnormal motor function of patients' upper limbs as well as their discontinuity of circle-drawing movements. This study indicates the muscle synergy analysis during the HRI with constrained circle-drawing movement could be considered as a task for upper-limb motor function assessments.

There are still several limitations in this study. Firstly, the sEMG signals are normalized to the peak value for a specific task [27]. However, the maximal isometric voluntary contraction (MVC) may not represent the real maximal activating level of muscles during the complex movements [28]. The MVC measurements in patients are usually affected by their varying degrees of motor deficits. This might bring a larger intersubject variability [29]. Nevertheless. the sEMG variations between different tasks and the same task collected at different recovery stages in the same patients could not be intuitively comparable by this normalization method [28]. In future study, a proper method of sEMG normalization is needed to be considered.

Secondly, the number of extracted muscle synergies has been proposed to reflect the complexity of motor control [16]. As mentioned in Methods, we extracted the number of muscle synergies by using VAF for all participants. A threshold needs to be set by experience. The thresholds may be different between healthy subjects and stroke patients. Therefore, a more objective approach to determine the number of muscle synergy is needed to be further developed.

Thirdly, due to the limited clinical resource, the sample size of stroke patients was only two in this study. The trend of decrease of muscle synergy number was found when the stroke patients were compared with healthy subjects, but there was no statistical evidence due to small sample size. A larger sample size of stroke patients with similar disease stage will be considered in the future study.

## Figures and Tables

**Figure 1:** Setup and experimental design. Participants were asked to keep their upper body stable, and their forearm was tied to the joystick of EULRR. (a) Participants sit on the left side of EULRR to implement circle-drawing movement by using their right hands; (b) the illustration of clockwise and counterclockwise circle-drawing movements with constraint of EULRR system.

**Figure 2:** The illustration of sEMG data preprocessing and muscle synergy analysis.

**Figure 3:** The typical sEMG results of six muscles in upper limb during the HRI with circle-drawing movements. (a) The sEMG results for counterclockwise circle-drawing movements; (b) the sEMG results for clockwise movements.

**Figure 4:** The comparison of raw and reconstructed sEMG data from factorized matrices.

**Figure 5:** The typical results of muscle synergies of upper limbs for healthy subjects during the HRI with counterclockwise circle-drawing movements. (a) The synergy pattern and activation coefficients for the first synergy; (b) the synergy pattern and activation coefficients for the second synergy; (c) the synergy pattern and activation coefficients for the third synergy. The structure of synergy represents the synergy pattern of muscle synergies, and the recruitment mode represents the activation coefficients of muscle synergies.

**Figure 6:** The typical results of muscle synergies of upper limbs for healthy subjects during the HRI with clockwise circle-drawing movements. (a) The synergy pattern and activation coefficients for the first synergy; (b) the synergy pattern and activation coefficients for the second synergy; (c) the synergy pattern and activation coefficients for the third synergy. The structure of synergy represents the synergy pattern of muscle synergies, and the recruitment mode represents the activation coefficients of muscle synergies.

**Figure 7:** The typical results of muscle synergies of upper limbs for stroke patients during the HRI with counterclockwise circle-drawing movements. (a) The synergy pattern and activation coefficients for the first synergy; (b) the synergy pattern and activation coefficients for the second synergy. The structure of synergy represents the synergy pattern of muscle synergies, and the recruitment mode represents the activation coefficients of muscle synergies.

**Figure 8:** The typical results of muscle synergies of upper limbs for stroke patients during the HRI with clockwise circle-drawing movements. (a) The synergy pattern and activation coefficients for the first synergy; (b) the synergy pattern and activation coefficients for the second synergy. The structure of synergy represents the synergy pattern of muscle synergies, and the recruitment mode represents the activation coefficients of muscle synergies.

## Data Availability

The (Excel) data used to support the findings of this study are available from the corresponding author upon request.

## Abbreviations

HRI: Human-robot interaction
sEMG: Surface electromyography
NMF: Nonnegative matrix factorization
EULRR: End-effector upper-limb rehabilitation robot
AD: Anterior deltoid
PD: Posterior deltoid
BB: Biceps brachii
TB: Triceps brachii
FCR: Flexor carpi radialis
ECR: Extensor carpi radialis
SENIAM: Surface EMG for noninvasive assessment of muscles
VAF: Variance account for
MVC: Maximal voluntary contraction.
